The article "Effect of Predictive Nursing Combined with Early Drinking Water Therapy on Patients with Urinary Retention after Vaginal Delivery" was published in 2022. Journal: Comput Math Methods Med.

# Effect of Predictive Nursing Combined with Early Drinking Water Therapy on Patients with Urinary Retention after Vaginal Delivery

**DOI:** 10.1155/2022/4204762

**Published:** 2022-06-30

**Authors:** Gaiying Cui, Yong Zhang, Zhaoxia Liu, Xia Li, Manting Sha

**Affiliations:** Shijiazhuang Fourth Hospital, China

## Abstract

The aim of this study is to analyze the effect of predictive nursing combined with early drinking water therapy on patients with urinary retention after vaginal delivery. A total of 600 women who gave birth in our hospital from July 2019 to July 2020 were selected as the research objects. A double-blind method was adopted to divide them into a control group and observation group, 300 cases in each group. In the control group, routine nursing was given. In the observation group, (1) predictive nursing measures were used before surgery. (2) The postoperative observation group used early drinking water therapy; the incidence of urinary retention, the effective rate of urination, postpartum haemorrhage, and the treatment of urinary retention were compared between the two groups. In the observation group, the number of urinary retention was 17, and the incidence of urinary retention was 5.67%. The urination efficiency of the observation group was 98.33%; the urination efficiency of the control group was 86.33%; comparison results showed that *P* < 0.05. The 24 h postpartum haemorrhage of the observation group was 1.33%; the 24 h postpartum haemorrhage of the control group was 2.66%. Uroschesis therapy was performed in 17 patients in the observation group and 44 patients in the control group.. The observation group had an 88.24 percent treatment rate, while the control group had a 72.73 percent treatment rate. *P* < 0.05 indicated that the difference was statistically significant.

## 1. Introduction

Postpartum retention refers to inability to urinate by oneself or inability to urinate properly for 6-8 hours after delivery, which is one of the common complications of postpartum [1]. It is a disease caused by bladder muscle paralysis caused by uterine pressure on bladder and pelvic nerve plexus during childbirth. Common reasons are being not used to urination in bed, sudden abdominal pressure, pain, psychological factor, and so on, which affect the recovery of patients after childbirth [2]. It has been reported in the literature that the incidence of postpartum urinary retention in vaginal delivery women is about 12~18% [3]. At present, there is no specific treatment to prevent and treat postpartum urinary retention. The traditional noninvasive method is induced urination, but its success rate is low [4, 5]. However, retention of urinary catheters can easily cause urinary tract infections. Studies have shown that urinary tract infections caused by urinary catheters account for 60% to 80% of patients with urinary tract infections. Effective clinical measures should be taken to prevent urinary retention [6, 7].

The article "Effect of Predictive Nursing Combined with Early Drinking Water Therapy on Patients with Urinary Retention after Vaginal Delivery" was published in 2022. Journal: Comput Math Methods Med.

Predictive nursing also known as advanced nursing takes preventive measures to reduce or avoid the occurrence of complications to a certain extent [8].

Studying on the effect of predictive nursing combined with early drinking water therapy on patients with urinary retention after vaginal delivery obtained good results. Predictive nursing combined with early drinking water therapy for the prevention and treatment of urine retention after vaginal delivery could effectively avoid urinary retention and improve the effective rate of urination. Expectant mothers should be encouraged to communicate with more experienced pregnant ladies.

The paper is arranged as follows: Section 2 discusses the materials and methods in detail.  Section 3 analyzes the experiments and result.  Section 4 concludes the article.

## 2. Materials and Methods

### 2.1. General Information

A total of 600 women who gave birth in our hospital from July 2019 to July 2020 were selected as the research objects. A double-blind method was adopted to divide them into a control group and observation group, 300 cases in each group. The control group 5was aged from 23 to 35, with an average age of 27.4. There were 180 parturient women, and the remaining 120 were parturient women; the observation group was 24 to 34 years old, with an average age of 27.2 years. There were 168 women who had already undergone parturition, and the remaining 132 were primiparous women. There was no statistically significant difference in general information between the two groups of patients (*P* > 0.05).

1. Diagnostic criteria: this refers to the diagnostic criteria for postpartum urinary retention in obstetrics and gynaecology in integrated traditional Chinese and Western medicine [9]. (1) 6 hours after delivery, urine dropped or became obstructed, and abdominal distension was acute and painful. (2) The lower abdomen was bulging, and the bladder was full and tender
2. Inclusion criteria: (1) primiparous women who gave birth vaginally <35 years old; (2) people with clear consciousness, able to cooperate with treatment, and without other diseases such as urinary tract infection; and (3) women who volunteered to participate in this trial and signed informed consent
3. Exclusion criteria: (1) having mental illness and unable to cooperate with the treatment, (2) combined with urinary system diseases, (3) severe postpartum complications, (4) persons with serious cardiopulmonary diseases, and (5) people with severe blood clotting disorder

The article "Effect of Predictive Nursing Combined with Early Drinking Water Therapy on Patients with Urinary Retention after Vaginal Delivery" was published in 2022. Journal: Comput Math Methods Med.

### 2.2. Methods

#### 2.2.1. Control Group

Routine care was given. Patients and their families are informed about the common clinical signs of postpartum urine retention. The difficulties to be handled prior to childbirth as well the importance of breastfeeding were explained. After childbirth, the nursing staff should understand the vaginal bleeding of the mother and understand whether she had urinated 6 hours after delivery.

#### 2.2.2. Observation Group

(1) Predictive nursing measures were used before surgery. In this group, predictive nursing measures were added, and the nursing content was as follows: (a) Physical status assessment: after admission, the patient's physical condition should be evaluated to understand the postpartum recovery of the patient. Under good condition, the patient could be assisted to get out of bed to urinate or raise the head of the bed to urinate on the bed. (b) Cognitive intervention: before giving birth, pregnant women should be informed of the causes of urinary retention and the importance of successful urination after surgery. Expectant mothers should be encouraged to communicate with more experienced pregnant ladies. Parturient women cooperated with medical staff to train and prevent postpartum urinary retention [10]. (c) Psychological intervention: medical staff should understand the psychological conditions of patients. Some maternal medical staff with fear and anxiety due to excessive worry should take appropriate measures to help the pregnant women stabilize their emotions, allowing women to have the best condition for surgery and gradually building up women's self-confidence in autonomous urination [11]. (4) In-bed urination training: medical staff needed to train the mother to urinate in bed and use toilets. This training was required three days before the operation. Training should be at least 2 to 3 times a day until the woman was ready to go to bed and defecate [12].

(2) The postoperative observation group was treated with early drinking water therapy. (a) Drinking water during labor: the puerpera is encouraged to drink water regularly and relieve urine once every 2~4 h. (b) Drinking water after delivery: during observation in the delivery room 2 h after delivery, the midwife guided the puerpera to water therapy in order to make the puerpera urinate as soon as possible. The specific methods are as follows: drinking 300~500 ml of warm water within 30 min after delivery, drinking 200~300 ml of warm water again 1 h after delivery, assisting the puerpera on their first pee by specially assigned personnel when the bladder is semifull or 1.52 h postpartum, and timely evaluation of bladder filling status during drinking water. (c) Urination training: while the patient was urinating, the medical staff could make the patient listen to the water to induce urination, and warm water could also be used to flush the perineum to stimulate urination. (d) Massage: the bladder area and uterus floor of the puerpera were massaged for 10 min/time, once every 0.5 h. The intensity was within the range of maternal tolerance. Massage action should not be too rough, and pay attention to the bladder area in the process of massage without swelling.

The article "Effect of Predictive Nursing Combined with Early Drinking Water Therapy on Patients with Urinary Retention after Vaginal Delivery" was published in 2022. Journal: Comput Math Methods Med.

### 2.3. Observational Index

The first urination and urine volume were recorded, and the volume of vaginal bleeding 24 hours after delivery was measured.

1. Incidence of urinary retention = number of cases of urinary retention/total cases × 100%
2. Effective rate of urination = (number of significant cases + number of effective cases)/total cases × 100%. The first urination volume > 500 ml was significant. The first urination volume of 100~500 ml was effective; the first urination volume < 100 ml was invalid
3. Postpartum haemorrhage: blood loss within 24 h after delivery is ≥500 ml
4. Uroschesis therapy: based on the bladder residual urine measured during the first and second urination after delivery and b-ultrasound after urination, the therapeutic effect of prevention of postpartum pigmentation was classified as special effect, obvious effect, effective, and invalid: special effects—urinary bladder residual urine volume ≤ 50 ml after urination within 2 h after delivery; obvious effect—the residual urine volume (≤50 ml) of the bladder after urination within 2-4 h after postpartum; effective—bladder residual urine volume ≤ 50 ml after urination within 4-6 h after postpartum; and invalid—those that did not meet the above criteria. For the first urination time > 6 hours, it was recorded as urinary retention and its incidence is counted

### 2.4. Statistical Methods

Using SPSS 22 statistical software, data were processed. Statistical data were compared by the *x*^2^ test. Measurement data were represented by *x* ± s, using the *t*-test. *P* < 0.05 meant that the difference was statistically significant.

## 3. Results

### 3.1. Results of the Incidence of Urinary Retention

In the observation group, the number of urinary retention was 17, and the incidence of urinary retention was 5.67%; in the control group, the number of urinary retention was 44, and the incidence of urinary retention was 14.67%. Results of the incidence of urinary retention are shown in Table 1.

### 3.2. Results of the Urination Efficiency

The urination efficiency of the observation group was 98.33%, and the urination efficiency of the control group was 86.33%; comparison results showed that *P* < 0.05. Results of the urination efficiency are shown in Table 2.

The article "Effect of Predictive Nursing Combined with Early Drinking Water Therapy on Patients with Urinary Retention after Vaginal Delivery" was published in 2022. Journal: Comput Math Methods Med.

### 3.3. Results of Postpartum Haemorrhage

The 24 h postpartum haemorrhage of the observation group was 1.33%; the 24 h postpartum haemorrhage of the control group was 2.66%. Results of postpartum haemorrhage are shown in Table 3.

### 3.4. Results of Uroschesis Therapy

Uroschesis therapy was performed in 17 patients in the observation group and 44 patients in the control group. The treatment rate in the observation group was 88.24%; the treatment rate of the control group was 72.73. The difference was statistically significant (*P* < 0.05). Results of urinary retention therapy are shown in Table 4.

Postpartum nervous tension and bladder compression during delivery can lead to bladder mucosa edema and congestion, decreased bladder muscle tension, or decreased pelvic pressure, resulting in urinary retention [13, 14]. Among the causes of patients with urinary retention, the main reasons are being unaccustomed to urinating in bed, sudden drop in abdominal pressure, pain, and psychological reasons [15]. At the same time, due to the lack of knowledge of postpartum health care, women and their families do not understand the importance of urinating as soon as possible after delivery. Inadequate or excessive drinking of water, failure to urinate regularly, and an overfilled bladder lead to urinary tract infections and increased rates of postpartum bleeding; thus, the recovery time of the patient's follow-up palmitis can be increased [16, 17]. Predictive nursing primarily uses health disease knowledge education and psychological intervention so that pregnant women can make appropriate preparations ahead of time, which can relieve the stress of patients entering the ward for the first time, establish harmonious medical care, and improve the pregnant women's trust and cooperation [18]. At the same time, the puerpera should be treated with drinking water therapy to make the puerpera feel like urinating as soon as possible. When the bladder is in a semifilled state or 1.5 to 2 hours after delivery, a person will help the puerpera to urinate, reducing the time it takes to urinate for the first time and recovering urinary function as soon as feasible [19, 20].

According to the findings, there were 17 cases of urine retention in the observation group, and the incidence of urinary retention was 5.67 percent; in the control group, the number of urinary retention was 44, and the incidence of urinary retention was 14.67%. The urination efficiency of the observation group was 98.33%, and the urination efficiency of the control group was 86.33%; comparison results showed that *P* < 0.05. The 24 h postpartum haemorrhage of the observation group was 1.33%; the 24 h postpartum haemorrhage of the control group was 2.66%. Uroschesis therapy was performed in 17 patients in the observation group and 44 patients in the control group. The treatment rate in the observation group was 88.24%; the treatment rate of the control group was 72.73. The difference was statistically significant (*P* < 0.05).

The article "Effect of Predictive Nursing Combined with Early Drinking Water Therapy on Patients with Urinary Retention after Vaginal Delivery" was published in 2022. Journal: Comput Math Methods Med.

## 4. Conclusion

To sum up, the application of predictive nursing combined with early drinking water therapy for the prevention and treatment of urinary retention after vaginal delivery could effectively prevent the occurrence of urinary retention after vaginal delivery and improve the effective rate of urination. It not only did not increase the incidence of postpartum haemorrhage at 2 h or 24 h but also improved the therapeutic effect of urination, and it was worth promoting.

## Figures and Tables

**Table 1:** Results of the incidence of urinary retention.

Groups	*n*	First urination time	Urination			
			0-4 h	4-6 h	Urinary retention	Incidence of urinary retention
Observation group	300	2.08 ± 1.02	274	9	17	5.67%
Control group	300	2.07 ± 1.41	231	25	44	14.67%

**Table 2:** Results of the urination efficiency.

Groups	*n*	Special effect	Obvious effect	Effective	Invalid
Observation group	300	90.0	205	5	98.333
Control group	300	73.1	186	41	86.333

**Table 3:** Results of postpartum haemorrhage.

Groups	*n*	2 h postpartum haemorrhage	24 h postpartum haemorrhage
Observation group	300	179.540 ± 12.161	4 (1.333)
Control group	300	18.533 ± 12.033	8 (2.662)

**Table 4:** Results of uroschesis therapy.

Groups	*n*	Special effect	Obvious effect	Effective	Invalid	Rate
Observation group	17	4	6	5	2	88.24%
Control group	44	8	13	11	12	72.73%

## Data Availability

The datasets used during the present study are available from the corresponding author upon reasonable request.
